The article "Clinical Characteristics of Diabetes Complicated by Bacterial Liver Abscess and Nondiabetes-Associated Liver Abscess" was retracted in 2023. Reasons: suspected computer-generated content; unreliable results or conclusions; concerns about the data; concerns about the results or conclusions.

# Clinical Characteristics of Diabetes Complicated by Bacterial Liver Abscess and Nondiabetes-Associated Liver Abscess

**DOI:** 10.1155/2022/7512736

**Published:** 2022-04-26

**Authors:** Fei Wang, Jingwen Yu, Wenjie Chen, Zewei Mo, Yuhai Zhang

**Affiliations:** Department of Endocrinology, Hainan General Hospital, Hainan Affiliated Hospital of Hainan Medical University, Haikou, Hainan 570311, China

## Abstract

**Background:**

Bacterial liver abscess (BLA) is a secondary infectious disease caused by hepatic parenchymal inflammation and bacterial necrosis. Studies have shown that diabetic patients with BLA have higher rates of related adverse events than patients without diabetes.

**Aim:**

To explore the clinical characteristics of BLA complicated with diabetes and nondiabetes-related BLA.

**Methods:**

From January 2019 to June 2020, 61 diabetic patients with BLA were included as the study group, and 61 BLA patients without diabetes were included as the control group. Clinical manifestations, laboratory examination index (prothrombin activity (PTA), albumin (propagated), white blood cell count (WBC), red blood cell count (RBC), plasma fibrinogen (FIB), C-reactive protein (CRP), neutrophil percentage (NEUT), and prealbumin (PA)) levels, blood cultivation, and fester situation in the two groups were analyzed.

**Results:**

No differences of Fever, right upper abdominal pain, jaundice, vomiting and nausea, liver tenderness, and liver pain upon percussion were observed between the study and control groups. However, chill, cough and expectoration, and liver pain upon percussion were higher in the study group, while abdominal distension was lower. WBC, RBC, PA, PTA, FIB, and CRP were higher than the control group. NEUT was higher in the study group than in the control group and Alb was lower than that in the control group. There was no significant difference between the positivity of blood bacterial culture in the study and control groups. The positivity rate of *Klebsiella pneumoniae* in Gram-negative aerobic bacteria in the study group was higher than that in the control group. There was no significant difference between the positivity of fester culture of the two groups. The positivity of *K. pneumoniae* in Gram-negative aerobic bacteria in the study group was higher than that in the control group. The positivity of *E. coli* was lower in the study group than in the control group.

**Conclusion:**

Clinical manifestations and laboratory results of BLA patients with and without diabetes mellitus were significantly different. The symptoms of diabetics with BLA were serious.

## 1. Introduction

Bacterial liver abscess (BLA) refers to an abscess caused by a liver parenchymal inflammatory response and necrosis to bacteria entering the liver in different ways and is known as a secondary infectious disease.

The article "Clinical Characteristics of Diabetes Complicated by Bacterial Liver Abscess and Nondiabetes-Associated Liver Abscess" was retracted in 2023. Reasons: suspected computer-generated content; unreliable results or conclusions; concerns about the data; concerns about the results or conclusions.

With the increasing morbidity of diabetes in recent years, the incidence of diabetes combined with BLA has also continued to increase, mainly because a chronic increase in blood glucose can cause an increased plasma osmotic pressure, leading to inhibition of leukocyte chemotaxis, phagocytosis, and adhesion resulting in lowered immunity. This is beneficial for bacterial multiplication and growth, resulting in hepatapostema, and a great threat to the quality of life, as well as the mental and physical health of patients [1–3].

Relevant statistical data have shown that, compared with BLA patients without diabetes, those with diabetes have approximately 3.6 times higher incidence of related hazardous events [4, 5]. Early diagnosis is essential for the treatment of the disease [6]. Therefore, it is of great significance to clarify the clinical characteristics of diabetic and nondiabetic patients complicated with BLA to guide the differential diagnosis of the disease and implement targeted treatment [7]. Thus, 61 diabetic and 61 nondiabetic patients with BLA were selected for a comparative study to clarify the differences in clinical characteristics between the two groups. The report is as follows.

## 2. Materials and Methods

### 2.1. Baseline Data

From our hospital, 61 patients with diabetes combined with BLA and 61 nondiabetic patients with BLA from January 2019 to June 2020 were selected as the study and control groups, respectively. There were 39 males and 22 females in the study group, with ages ranging from 34 to 79 years, with an average of 56.45 ± 9.06 years. The duration of diabetes was 1.5–13.5 years, with an average of 7.50 ± 2.35 years. The lesion size was 3.3–11.6 cm, with an average of 7.45 ± 3.07 cm. Meanwhile, there were 36 males and 25 females in the control group with an average age of 55.39 ± 8.22 years, ranging from 31 to 79 years old. The lesion size ranged from 3.1 cm to 12.2 cm, with an average of 8.01 ± 2.96 cm. The clinical data of the two groups were equally comparable (*P* > 0.05), and the study was approved by the ethics committee of our hospital.

## 3. Selection Criteria

### 3.1. Inclusion Criteria

The inclusion criteria were as follows: (1) Hepatapostema was clearly diagnosed through MRI, CT, or B ultrasound examination, (2) patients and their families provided informed consent for the study, (3) diagnosis was achieved by percutaneous hepatocentesis, and (4) patients had good compliance and could cooperate to complete the investigation.

### 3.2. Exclusion Criteria

The exclusion criteria were as follows: (1) Patients with liver liquefaction infarction, liver echinococcosis, tuberculous liver abscess, and amoeba liver abscess, (2) patients with leukemia, nephrotic syndrome, and end-stage renal disease; (3) presence of abdominal abscess; (4) liver tumor; (5) verbal communication disorders, cognitive dysfunction, and mental system diseases; (6) patients with blood system diseases; and (7) other acute and chronic infectious diseases.

The article "Clinical Characteristics of Diabetes Complicated by Bacterial Liver Abscess and Nondiabetes-Associated Liver Abscess" was retracted in 2023. Reasons: suspected computer-generated content; unreliable results or conclusions; concerns about the data; concerns about the results or conclusions.

## 4. Methods

(1) The clinical manifestations of the two groups were assessed, such as fever, right upper abdominal pain, jaundice, vomiting and nausea, liver tenderness, pain in the liver area upon percussion or palpation, chills, abdominal distention, and cough and sputum. (2) The laboratory test indexes of the two groups were measured, including prothrombin activity (PTA), albumin (Alb), white blood cell count (WBC), red blood cell count (RBC), plasma fibrinogen (FIB), C-reactive protein (CRP), neutrophil percentage (NEUT), and prealbumin (PA) levels. PTA and FIB were determined using a Pulisson C3510 automatic coagulation analyzer (Japan Xisen Micon Medical Electronics Co., Ltd.), and Alb was determined using an AU400 automatic biochemical analyzer (Beckman Coulter Company, USA). WBC, RBC, PA, and NEUT were determined using a BC5390 hematology analyzer (Japan Hisen Micon Medical Electronics Co., Ltd.). CRP was determined using an enzyme-linked immunosorbent assay (ELISA) with a Bio-Rad 550 ELISA kit. (3) Blood culture and fester culture were done by collecting venous blood and fester and placing them in culture bottles. These were cultured in a BACT/ALERT 3D 60 automatic blood culture instrument, and VITEK 2-Compact 60 automatic bacteria identification and drug sensitivity analysis were used for microbial identification

### 4.1. Observation Indexes

(1) The clinical manifestations of the two groups were assessed. (2) The levels of laboratory examination indices of the two groups were statistically analyzed. (3) Blood cultures of the two groups were assessed. (4) The statistics of the two groups of pus cultures were analyzed

### 4.2. Statistical Analysis

SPSS22.0 was used for data analysis. Measurement data were expressed as ±s, independent sample *t*-test was used for intergroup comparison, paired *t*-test was used for intragroup comparison, count data were expressed as cases (%), and *χ*^2^ test was used. Statistical significance was set at *P* < 0.05.

## 5. Results

### 5.1. Comparison of Clinical Manifestation between the Two Groups

No significant difference was noted in fever (98.36%), right upper abdominal pain (42.62%), jaundice (6.56%), vomiting and nausea (19.67%), liver tenderness (19.67%), and pain upon palpation or percussion of the liver (6.56%) in the study group than in the control group (93.44%, 47.54%, 13.11%, 14.75%, 27.87%, and 9.8%, respectively (*P* > 0.05). Chills (73.77%), cough and expectoration (18.03%), and liver tenderness and pain upon palpation or percussion (19.67%) were higher in the study group than in the control group (54.10%, 3.28%, and 4.92%), and abdominal distension (1.64%) was lower than that in the control group (19.67%) (*P* < 0.05). These results are shown in Table 1.

The article "Clinical Characteristics of Diabetes Complicated by Bacterial Liver Abscess and Nondiabetes-Associated Liver Abscess" was retracted in 2023. Reasons: suspected computer-generated content; unreliable results or conclusions; concerns about the data; concerns about the results or conclusions.

### 5.2. Comparison of Laboratory Examination Indices between the Two Groups

WBC (14.67 ± 8.61) ×10^9^/L, RBC (3.73 ± 0.65) ×10^12^/L, PA (68.98 ± 10.04) mg/L, PTA (75.69 ± 13.64)%, FIB (6.37 ± 1.51) g/L, and CRP (96.60 ± 33.85) mg/L levels were higher in the study group than those in the control group (WBC (12.91 ± 6.99) ×10^9^/L, RBC (3.68 ± 0.70) ×10^12^/L, PA (71.15 ± 12.33) mg/L, PTA (77.35 ± 12.83)%, FIB (6.69 ± 1.72) g/L, and CRP (99.91 ± 29) mg/L. NEUT (85.25 ± 6.61)% in the study group was higher than that in the control group (78.96 ± 7.20)%, and Alb (27.25 ± 3.54) g/L was lower than that in the control group (30.91 ± 4.01) g/L (*P* < 0.05). These results are shown in Table 2.

### 5.3. Comparison of Blood Culture between the Two Groups

There was no significant difference between the positive rate of blood bacterial culture in the study group (77.05%) and that in the control group (59.02%) (*P* > 0.05), and the positivity of *Klebsiella pneumoniae* in Gram-negative aerobic bacteria in the study group (63.93%) was higher than that in the control group (37.70%) (*P* < 0.05). These results are shown in Table 3.

### 5.4. The Comparison of Fester Cultivation between the Two Groups

There was no significant difference between the positivity of fester culture in the study group (96.72%) and the control group (88.52%) (*P* > 0.05). The positivity of *K. pneumoniae* in Gram-negative aerobic bacteria in the study group (81.97%) was higher than that in the control group (52.46%). The positivity of *E. coli* (4.92%) was lower than that of the control group (18.03%) (*P* < 0.05). These results are shown in Table 4.

## 6. Discussion

Chronically increased blood glucose levels in diabetic patients can cause increased plasma osmotic pressure, leading to inhibition of leukocyte chemotaxis, phagocytosis, and adhesion, and decreasing immunity. In addition, most patients with diabetes have certain vascular lesions, resulting in slow blood flow speed, which can further hinder the mobilization and movement of WBC, leading to diabetes patients becoming a high-risk group of BLA.^[^ [8–10]^]^ Statistical data showed that the risk of BLA in diabetic patients is approximately 3.6–11 times higher than that in healthy people, but there are differences in reports from different regions. The incidence of diabetes with BLA is high in Asian countries, ranging between 26% and 56.8%, while the incidence is low in Western countries [11–13]. In recent years, with the formation of bad living habits and the transformation of dietary patterns, the incidence of diabetes and the prevalence of diabetic patients with BLA have increased with most patients having no typical adverse signs and clinical symptoms, which has resulted in high misdiagnosis and missed diagnosis rates. If the patient does not receive timely effective intervention, the abscess will pierce the tissues and organs around the liver, resulting in empyema, subphrenic abscess, etc., or cause metastatic infections, including kidney abscess, lung abscess, and brain abscess, and then septic shock, sepsis, or even pose a threat to the life and health of the patient [8, 13, 14]. Therefore, it is of great significance to clarify the difference between BLA in diabetes mellitus patients and non-BLS diabetes mellitus patients, as a guide for the accurate differential diagnosis of BLA in diabetes mellitus and to guide targeted treatment.

The article "Clinical Characteristics of Diabetes Complicated by Bacterial Liver Abscess and Nondiabetes-Associated Liver Abscess" was retracted in 2023. Reasons: suspected computer-generated content; unreliable results or conclusions; concerns about the data; concerns about the results or conclusions.

Our study showed that the main clinical manifestation of patients with diabetes complicated with BLA is chills; abdominal pain may not be obvious as most patients with diabetes have different degrees of vasculopathy and neuropathy, and the body's sensitivity to pain is reduced. Meanwhile, patients with diabetes complicated with BLA have nonspecific clinical manifestations, such as coughing and expectoration, which can easily lead to misdiagnosis or missed diagnosis. Therefore, patients with unexplained right upper abdominal pain, chills, and fever should be suspected of having BLA, and the relevant examinations should be done to avoid related adverse events, especially in those with diabetes because of their low sensitivity to pain [15–17]. In the laboratory, the main indicators were electrolyte disorder, prolonged coagulation time, decreased albumin content, increased aminotransferase, anemia, increased neutrophil percentage, white blood cell count, etc. There were no significant differences in most indicators between the groups, but NEUT in the study group was higher than that in the control group (*P* < 0.05). This may be due to a more severe inflammatory response in patients with diabetes combined with BLA. The Alb level in the analysis group was lower than that in the control group because of the lack of insulin in diabetic patients, which further affects protein metabolism and synthesis [18, 19].

The article "Clinical Characteristics of Diabetes Complicated by Bacterial Liver Abscess and Nondiabetes-Associated Liver Abscess" was retracted in 2023. Reasons: suspected computer-generated content; unreliable results or conclusions; concerns about the data; concerns about the results or conclusions.

In recent years, the etiology of BLA has changed, and *K. pneumoniae* has become the dominant pathogen that mainly engrafts in the respiratory and digestive tracts of the healthy population. Usually, they are considered conditional pathogenic bacteria; however, if the body's immune function is decreased, intestinal barrier function injury can occur, which can cause a shift in the *K. pneumoniae* flora balance, resulting in infection. Some scholars confirmed that the positivity of *K. pneumoniae* in the blood culture and pus culture of patients with diabetes complicated with BLA was 60.27% and 82.78%, respectively, which is significantly higher than that of patients without diabetes complicated with BLA alone [20]. In this study, the blood cultivation and fester *K. pneumoniae* positivity in the study group was higher than that in the control group (*P* < 0.05), which was consistent with the results of a previous study. This may be attributed to impairment of the immune function of diabetic patients with BLA and can result in high plasma osmotic pressure. Additionally, high blood glucose can cause mononuclear phagocyte and neutrophil deformation and damage to consumption, adhesion, and chemotaxis function can occur. Thus, antibody production is reduced, and the patient develops a defect in the intima of the blood vessels, resulting in the spread of *K. pneumoniae* through the blood.

## 7. Conclusion

In conclusion, the clinical manifestations and laboratory results of BLA patients with diabetes mellitus and nondiabetes mellitus were significantly different, and the infection symptoms of patients with diabetes mellitus and BLA patients were serious. Furthermore, the infection rate of *K. pneumoniae* was higher, which should be the focus of future clinical research.

## Figures and Tables

**Table 1:** Comparison of clinical manifestation between the two groups (*n* (%)).

Groups	Cases	Fever	Right upper abdominal pain	Jaundice	Vomiting and nausea	Liver tenderness	Liver pounding pain	Chills	Cough and expectoration	Liver tenderness + knock pain	Abdominal distension
The study group	61	60 (98.36)	26 (42.62)	4 (6.56)	12 (19.67)	12 (19.67)	4 (6.56)	45 (73.77)	11 (18.03)	12 (19.67)	1 (1.64)
The control group	61	57 (93.44)	29 (47.54)	8 (13.11)	9 (14.75)	17 (27.87)	6 (9.84)	33 (54.10)	2 (3.28)	3 (4.92)	12 (19.67)
*Χ* ^2^ value		1.877	0.298	1.479	0.518	1.131	0.436	5.119	6.974	6.157	10.418
*P* value		0.171	0.585	0.224	0.472	0.288	0.509	0.024	0.008	0.013	0.001

**Table 2:** Comparison of the laboratory examination index between the two groups ($\bar{x}\pm s$).

Groups	Cases	WBC (×10^9^/L)	RBC (×10^12^/L)	PA (mg/L)	PTA (%)	FIB (g/L)	CRP (mg/L)	NEUT (%)	Alb (g/L)
The study group	61	14.67 ± 8.61	3.73 ± 0.65	68.98 ± 10.04	75.69 ± 13.64	6.37 ± 1.51	96.60 ± 33.85	85.25 ± 6.61	27.25 ± 3.54
The control group	61	12.91 ± 6.99	3.68 ± 0.70	71.15 ± 12.33	77.35 ± 12.83	6.69 ± 1.72	99.91 ± 29.97	78.96 ± 7.20	30.91 ± 4.01
*T* value		1.239	0.409	1.066	0.672	1.092	0.572	5.026	5.344
*P* value		0.218	0.683	0.289	0.503	0.277	0.569	0.000	0.000

The article "Clinical Characteristics of Diabetes Complicated by Bacterial Liver Abscess and Nondiabetes-Associated Liver Abscess" was retracted in 2023. Reasons: suspected computer-generated content; unreliable results or conclusions; concerns about the data; concerns about the results or conclusions.

**Table 3:** Comparison of blood cultivation situation between the two groups (*n* (%)).

Bacterial type	The study group (*n* = 61)	The control group (*n* = 61)	*χ* ^2^ value	*P* value
Positive rate of bacterial culture	47 (77.05)	36 (59.02)	4.560	0.033
Gram-negative aerobic bacteria				
Pseudomonas aeruginosa	1 (1.64)	1 (1.64)	0.000	1.000
Proteusbacillus vulgaris	1 (1.64)	3 (4.92)	1.034	0.309
Escherichia coli	2 (3.28)	4 (6.56)	0.701	0.402
Klebsiella pneumoniae	39 (63.93)	23 (37.70)	8.396	0.004
Gram-positive aerobic bacteria				
Enterococcus	2 (3.28)	1 (1.64)	0.342	0.559
Streptococcus	1 (1.64)	3 (4.92)	1.034	0.309
Staphylococcus aureus	1 (1.64)	1 (1.64)	0.000	1.000

**Table 4:** Comparison of fester cultivation situation between the two groups (*n* (%)).

Bacterial type	The study group (*n* = 61)	The control group (*n* = 61)	*χ* ^2^ value	*P* value
Positive rate of bacterial culture	59 (96.72)	54 (88.52)	3.000	0.083
Gram-negative aerobic bacteria				
Pseudomonas aeruginosa	1 (1.64)	2 (3.28)	0.342	0.559
Proteusbacillus vulgaris	1 (1.64)	2 (3.28)	0.342	0.559
Escherichia coli	3 (4.92)	11 (18.03)	5.164	0.023
Klebsiella pneumoniae	50 (81.97)	32 (52.46)	12.051	0.001
Gram-positive aerobic bacteria				
Enterococcus	2 (3.28)	1 (1.64)	0.342	0.559
Streptococcus	1 (1.64)	3 (4.92)	1.034	0.309
Staphylococcus aureus	1 (1.64)	3 (4.92)	1.034	0.309

## Data Availability

The authors confirm that the data supporting the findings of this study are available within the article.
